# Unilateral False Cord Nodule Presenting As Hoarseness in a Young Patient

**DOI:** 10.7759/cureus.40491

**Published:** 2023-06-16

**Authors:** Noorain N Muslim, Burhanuddin Salim, Santhi Kalimuthu, Shashi Gopalan, Mawaddah Azman

**Affiliations:** 1 Otolaryngology - Head and Neck Surgery, Universiti Kebangsaan Malaysia, Kuala Lumpur, MYS; 2 Otolaryngology - Head and Neck Surgery, Hospital Tengku Ampuan Rahimah, Klang, MYS

**Keywords:** vocal cord lesion, hoarseness, larynx, benign, false cord nodule

## Abstract

Vocal cord nodules are benign laryngeal lesions seen in professional voice users. They are usually bilateral and are thought to occur due to submucosal edema and hemorrhage, with resultant fibrosis. False cord occurrences are very rare; hence we report a unique case of unilateral right false cord nodule. A healthy 16-year-old female student presented with persistent hoarseness for two years without any history of voice abuse, trauma, infection, or endotracheal intubation. Endoscopic examination showed a mass occupying the right false cord. Subsequent direct laryngoscopy revealed a friable mass on the right false cord without any true cord involvement. Complete excision was done. Post-operatively her symptoms completely resolved, and flexible endoscopic examination seven months post-op showed no recurrence. Histopathological examination revealed fragments of fibro collagenous tissue covered by benign respiratory epithelium, favoring the diagnosis of a benign nodule. False cord benign lesions are rare. In a symptomatic case, endolaryngeal microsurgery gives a good outcome.

## Introduction

Benign vocal cord lesions include nodules, polyps, and cysts. Nodules commonly occur at the mid-membranous vocal cord, where maximal impact stress happens during phonation [1]. Voice abuse, overuse, and misuse lead to repeated mechanical trauma to this area, resulting in wound formation. The resultant fibrosis occurring at the superficial lamina propria causes hoarseness associated with these conditions [1]. While vocal cord lesions have been extensively studied in the literature, limited information is available on benign false cord lesions. We report a case of a unilateral false cord benign nodule.

This article was previously presented as a poster at the 11TH Malaysian International ORL-HNS Congress & 39th Annual General Meeting of the MSO-HNS on June 20, 2019.

## Case presentation

A healthy 16-year-old female student presented to the otorhinolaryngology clinic with a two-year history of hoarseness. There was no fever or weight loss, and her symptom was not associated with any breathing or swallowing difficulty. There was no history of preceding dental trauma, infection, or foreign body ingestion, and she had never been hospitalized prior to this. She was not a professional voice user, nor was there any history of preceding voice abuse. Perceptual voice evaluation showed overall dysphonia grade three with main components strain and rough voice.

Examination of the neck revealed no lymphadenopathy, and flexible endoscopic nasopharyngolaryngoscopy showed a mass at the right false cord, obscuring the view of the right true cord.

Subsequent direct laryngoscopy confirms a friable right false cord mass (Figure 1); however, vocal cords and subglottic area were both normal on examination. The mass was completely excised using cold instruments (Figure 2).

**Figure 1:** Direct laryngoscopic finding of the larynx noted right unilateral false cord nodule obscuring right true cord visualization (white arrow)

**Figure 2:** Intraoperative image showing a direct laryngoscopic view of completely excised right false cord lesion with normal vocal cord and subglottic area

The patient recovered uneventfully in the postoperative period, with marked improvement in her voice. Postoperative endoscopic examination in the clinic showed some granulation on the right false cord, which healed well seven months after, with only a mild bulge at the operated site.

The histopathological section of the mass shows multiple fragments of fibro collagenous tissue partly covered by benign respiratory-type epithelium (Figure 3).

**Figure 3:** Fragments of fibro collagenous tissue partly covered by benign respiratory-type epithelium (Hematoxylin and eosin staining, 20x)

The tissue was eosinophilic and hypocellular with mild lymphoplasmacytic cell infiltrate. A cluster of *Actinomyces spp* colony was seen, and Congo Red stain was negative for amyloid deposition.

## Discussion

Benign vocal cord lesions are thought to result from mechanical stress, in which voice abuse, overuse, and misuse lead to repeated mechanical trauma to this area, resulting in wound formation. Wound healing results in the remodeling of the superficial lamina propria, encompassing hyalinization and fibrosis, leading to increased stiffness with resultant hoarseness. Diagnosis of such lesions involves thorough medical and voice history, examination of the head and neck, perceptual assessment of the voice, and detailed imaging of the vocal cords. Laryngeal videostroboscopy remains the most practical and clinically useful tool in assessing vocal cord vibratory characteristics and glottal configuration, in which nodules tend to appear as white to opaque, symmetric, fusiform, and firm. They result in an hourglass closure glottal configuration and will affect the vocal cord mucosal wave and vibration variably [1].

On the contrary, false cord benign lesions are rare, in most part due to the obscurity of their precise anatomy and function. To the author's knowledge, there has only been one published case report on false cord nodules; unfortunately, the original author of the report was uncontactable for further details and comparisons [2].

While the vocal cords are known to directly contribute to phonation and protection of the lower airways, the anatomy nor the role of the false cords on phonation has not been clear in the literature, whereby their primary function was thought to take the role of a "valve" regulating the pressure between thoracic and intraabdominal cavity [3]. However, a cadaveric study on unilateral vocal cord palsy showed significant ipsilateral atrophy of the ventricularis and thyroarytenoid muscle (which make up the false cord) on the side with vocal cord palsy, suggesting a more prominent role of the false cord on normal phonation [3]. Consequently, the false cords may, in fact, be at risk of the same mechanical stress from voice abuse that affects the true cords, resulting in benign lesions such as a nodule.

First-line treatment for benign vocal cord lesions involves speaking and singing therapy to maximize the efficiency of the voice mechanism and reduce vibratory trauma to the cord. Additionally, treatment of poor vocal hygiene and laryngopharyngeal reflux also contributes to a positive outcome, especially in terms of perceptual improvement [1]. Surgical treatment may be undertaken if maximal behavioral intervention does not achieve satisfactory improvements. Laryngeal microsurgery has been shown to consistently produce good outcomes by means of improved perception, videostroboscopy findings, and aerodynamic measures [1].

In this patient's specimen, a cluster of actinomyces colonies was observed (Figure 3). Actinomycosis is a rare infection caused by the filamentous Gram-positive bacilli *Actinomyces spp*, of which *Actinomyces israelii* is the most prevalent in humans [4]. While they are frequently found as commensals in the oropharynx, gastrointestinal tract, and urogenital tract, *Actinomyces spp* usually possess low pathogenicity as they are saprophytes and are thought to only cause infection in the event of antecedent tissue injury by way of mucosa breach [5,6]. As actinomycoses tend to occur at different parts of the body, their presentation varies greatly. The cervicofacial form of actinomycoses, which encompasses head and neck involvement, is commonly found in the submandibular and parotid glands and the mandible [7]. Laryngeal involvement is rare. In our case, while there was a colony of actinomyces seen in the histopathologic examination, it was concluded by the reporting pathologist as not significant as there was an absence of surrounding peripheral inflammatory reaction. The most likely explanation for such findings would be the migration of the colony from the laryngeal instruments used during the procedure.

## Conclusions

This case report describes a rare occurrence of a unilateral right false cord nodule in a young patient presenting with persistent hoarseness. The diagnosis of vocal cord nodules is typically associated with professional voice users and bilateral involvement. However, this case report highlights the importance of considering false cord nodules in the differential diagnosis of hoarseness, even in the absence of voice abuse or other contributing factors. The increasing discovery of the false cord's role in normal phonation may explain the possible etiology of this condition.
